The article "HER4 Promotes Osteosarcoma Progression and Predicts Poor Prognosis through the PTEN-PI3K/AKT Pathway" was retracted in 2025. Reason: duplicated images.

# HER4 Promotes Osteosarcoma Progression and Predicts Poor Prognosis through the PTEN-PI3K/AKT Pathway

**DOI:** 10.7150/jca.62787

**Published:** 2022-01-01

**Authors:** Kun Ma, Chuan Zhang

**Affiliations:** Luoyang Orthopaedic Hospital of Henan Province & Orthopaedic Hospital of Henan Province, Luoyang, Henan 471002, China.

**Keywords:** HER4, osteosarcoma, invasion, stemness trait, PTEN, PI3K/mTOR pathway

## Abstract

Studies have reported a relationship between human epidermal growth factor receptor 4 (HER4), a ubiquitously expressed and unique member of the ErbB family, and clinicopathological features of osteosarcoma. However, further investigation is warranted. HER4 expression was analyzed by quantitative reverse transcription-polymerase chain reaction, western blotting, and immunohistochemistry. The relationship between HER4 expression and the prognosis of patients with osteosarcoma was determined by constructing a Kaplan-Meier curve. Cell viability and proliferation were investigated by MTT and colony formation assays. The mechanism underlying HER4-modulated proliferation and invasion/migration of osteosarcoma cells was determined by short hairpin RNA (shRNA) interference, colony formation, migration, invasion, and western blotting experiments. Spheroid formation assay and CD133+ cell populations were used to examine HER4-induced stem-like traits.

The present findings revealed that HER4 was overexpressed in both osteosarcoma cells and tissues. Moreover, this overexpression was associated with high Enneking stage, metastasis, and recurrence. Sh-HER4 showed obviously suppressed cell viability, colony formation, and invasion/migration. In addition, knockdown of HER4 markedly attenuated the spheroid size and proportion of CD133-positive cells, as well as the expression of stemness markers. Sh-HER4 also reduced the tumor size, downregulated the expression of phosphorylated-PI3K (p-PI3K) and p-AKT, and increased that of p-phosphatase and tensin homolog (p-PTEN) in mouse tissue. From a mechanistic perspective, HER4 knockdown activated p-PTEN and suppressed p-PI3K and p-AKT expression. HER4 promoted osteosarcoma progression through inactivation of the PTEN-PI3K/AKT pathway.

Taken together, the results indicate that HER4 represents a novel target in osteosarcoma progression and stemness modulation, and may be of value for the development of treatments against osteosarcoma.

## Introduction

Osteosarcoma, the most common primary malignant bone tumor, which occurs in children and adolescents 1, is characterized by spindle stromal cells that directly form bone tissue 2. Although adjuvant and neo‑adjuvant chemotherapy have been introduction in the past decade, the majority (50-60%) of patients with osteosarcoma have advanced or metastatic disease by the time of diagnosis 3-4. The identification of reliable and effective prognostic biomarkers for osteosarcoma is an urgent challenge and target for clinical research.

HER4 is a ubiquitously expressed and unique member of the ErbB family 5. High levels of EGFR are found in 50-70% of lung 6, colon 7, and breast 8 carcinomas, and are considered to promote cell viability 9, cell cycle progression 10, and survival 11; in addition, they are associated with poor prognosis in patients with cancer 12. Some research studies have investigated the relationship between HER4 levels and progression of osteosarcoma 13. However, these findings are unilateral and fragmentary. To date, there are no comprehensive systematic studies of the effects of HER4 hyperactivation on tumorigenesis and disease aggressiveness in this type of cancer.

Phosphatase and tensin homolog (PTEN) deleted on chromosome 10 was the first tumor suppressor gene with tyrosine phosphatase activity to be discovered 14. Several studies have demonstrated that PTEN regulates cancer stem cells and epithelial-to-mesenchymal (EMT) transition via the PI3K/AKT pathway in glioma 15, lung cancer 16, and pancreatic cancer 17. Studies also have also shown that the AKT/mechanistic target of rapamycin kinase (AKT/mTOR) pathway is involved in the development of osteosarcoma 18-21.

The aim of this study was to investiage whether HER4 represents a promising novel therapeutic target for the prevention of metastasis and a potential prognostic biomarker for patients with osteosarcoma. We examined, in detail, the relationship between HER4 expression and clinicopathological features and prognosis of patients with osteosarcoma. Furthermore, the biological roles of HER4 knockdown on cell proliferation, invasion/migration, EMT, and modulation of stemness traits as well as the molecular basis for such effects, were also characterized. The present findings demonstrated that HER-4 may serve as an oncogene in osteosarcoma development and progression, recommending HER-4 as a promising prognostic marker and therapeutic target forosteosarcoma.

## Materials and Methods

### Tissue samples

Osteosarcoma tissues were collected from patients (41 men and 34 women) who were diagnosed with osteosarcoma and had undergone surgery between 2013 and 2018. Inclusion criteria: (1) All patients were confirmed as osteosarcoma during operation. (2)No radiotherapy, chemotherapy or immunotherapy was received before surgery. (3) The clinical information is complete. Exclusion criteria: (1) complicated with other malignant tumors. (2) Some patients were transferred in the course of treatment. (3) Patients who do not cooperating with research. The average age of the patients was 33 years (range: 16-38 years). The following information was obtained: sex, age, tumor size, clinical stage, tumor location, lung metastasis, and recurrence status. None of the patients had received other treatments (e.g., chemotherapy or radiotherapy) prior to surgery.Hematoxylin- and eosin-stained sections were independently diagnosed by two pathologists using the World Health Organization classification for osteosarcoma. The study were approved by the Medical Ethics Committee of Luoyang Orthopaedic Hospital of Henan Province and Orthopaedic Hospital of Henan Province (Luoyang, China). Written informed consent was provided by all the participants.

### Cell culture and reagents

Human osteosarcoma cells (U2OS, MG-63, HOS, and SaoS2 cells) were obtained from the Shanghai Institute of Biochemistry and Cell Biology (Chinese Academy of Sciences, Shanghai, China) and cultured in RPMI‑1640 or DMEM medium containing 10% fetal bovine serum (FBS) and placed in a 5% CO2 incubator at 37°C. The osteoblastic human fetal osteoblast (hFOB) 1.19 cells were seeded in Dulbecco's modified Eagle's medium/F-12 containing 10% FBS and 0.3 mg/mL of geneticin.

### Groups

The following 10 groups, which were divided into three stages, were analyzed: Stage I: sh-control group; sh-HER4 group; Stage II: sh-control; sh-HER4 group; LY294002 group; sh-HER4+LY294002 group; 25 μM LY294002 which was obtained from Abcam (cat. no. ab146593; Abcam, Cambridge, UK) was added to inhibit the activation of the PI3K/AKT pathway. Stage III: sh-control group; sh-HER4 group; sh-PTEN group; sh-HER4+sh-PTEN group.

### MTT assay

The *in vitro* cell proliferation was examined by MTT assay. After transfection with sh-control or sh-HER4 for 24, 48, and 72 h, U2OS and MG-63 cells were maintained in 96-well flat-bottom microtiter plates overnight at 4˚C. The supernatant was discarded, and the plates were washed three times with tap water and air dried.Subsequently, 20 μL of MTT solution was added to the cells, followed by incubation for 4 h at 37°C. The absorbance was measured at 570 nm using an automatic multi-well spectrophotometer.

### Sphere formation assay

The indicated cells (control cells and HER-4 knockdown cells) were cultured in growth medium containing 1% N2 serum-free cell culture additives, 2% B27 serum-free cell culture supplement (Gibco; Thermo Fisher Scientific, Inc.), 20 ng/mL of human platelet growth factor and so on in a humidified incubator under 5% CO2 at 37°C. After culturing 10 days, Sphere sizes were subsequently assessed using an inverted microscope.

### Fluorescence-activated cell sorter analysis

Osteosarcoma cells were blocked and suspended at 0°C for 15 min. Next, cells were labelled with phycoerythrin anti-human CD133 antibody for 60 min, washed twith PBS for two times, and maintained at 0°C until analysis. The expression of CD133 was analysed by Flow cytometry (FACS Calibur; BD Bioscience, USA).

### Western blotting

Western blotting was performed as previously described. Cells were washed and re-suspended at 25°C. Following treatment for 30 min, cell lysates were centrifuged at 14,000 × *g* at 4 °C. The primary antibodies are used at the manufacturer's recommended dilution: phosphorylated-PI3K (p-PI3K), p-AKT, p-PTEN, caspase-3(CASP3), glyceraldehyde-3-phosphate dehydrogenase (GAPDH), alpha-smooth muscle actin (α-SMA), E-cadherin, vimentin, NANOG, octamer-binding transcription factor 4 (Oct4), and SRY-box transcription factor 2 (SOX2). Finally, secondary antibodies (1:5,000 dilution) were added to the membranes at 25°C for 2 h. GAPDH was used as a loading control.

### Transwell assay

For the invasion assay, transwell chamber embedded with matrigel was employed. Indicated cells were cultured for 48 h under the same conditions. Finally, cells that invaded into the lower chambers were fixed for 30 min in 4% formaldehyde and stained for 15 min, took photos with an inverted phase-contrast microscope.

### Wound closure assay

Cells were seeded in fixed medium supplemented with 10% FBS. Then various treatments were performed while cells' confluent reached to 70%.After washing with PBS for three times, the wounds were monitored at 0 and 48 h using the Cell Imaging System (Zeiss GmbH). The wound healing data were taken at 0 h and 48 h using the Eclipse TE-2000-u inverted microscope (Nikon).

### HER4 knockdown

shRNA#1, shRNA#2, and shRNA#3 for HER4 were designed and synthesized by Genechem Company. When the confluence of U2OS and MG-63 cells in the six-well plate reached 50%, the cells were transfected with HER4 shRNA#1, shRNA#2, shRNA#3, or negative control. Subsequently, the cells were incubated for 48 h, and the expression levels of HER4 were determined by western blotting. HER4-#1 sense 5'-GATCCGCATTGGCACAGGATCATTGATTCAAGAGATCAATGATCCTGTGCCAATGCTTTTTTG-3', antisense 5'-AATTCAAAAAAGCATTGGCACAGGATCATTGATCTCTTGAATCAATGATCCT GTGCCAATGCG-3'; HER4 #2 sense 5'-GATCCGGTCCTGACAACTGTACAAAGTTCAAGAGACTTTGTACAGTTGTCAGGACCTTTTTTG-3', antisense 5'-AATTCAAAAAAGGTCCTGACAACTGTACAAAGTCTCTTGAACTTT GTACAGTTGTCAGGACC G-3'; HER4 #3 sense 5'-GATCCGCTCTTCATTCTGGTCATTGTTTCAAGAGAACAATGACCAGAATGAAGAGCTTTTTTG-3', antisense 5'-AATTCAAAAAAGCTCTTCATTCTGGTCATTGTTCTCTTGAAACAATGACCAGAATGAAGAGCG-3'; sh-control sense 5'-GATCCCGCAAACCCATGATTTACATTCAAGAGATGTAAATCATGGGATGGGATTTGCTTTTTA-3, antisense 5'-AGCTTAAAAGCAAATCCCATGATTTACATCTCTTGAATGTAAATCATGGGATTTGC-3'.

### Quantitative reverse transcription-polymerase chain reaction (qRT-PCR) analysis

The tissues were extracted and fragmented. A PCR detection system (Thermo, ABI 7500, USA) was used to detect the expression of human epidermal growth factor receptor 4. All experiments were executed in line with the instructions provided by the manufacturer. GAPDH was used as the internal control for gene expression. The primer sequences were as follows: HER4 forward: 5'-TTTCAAGGGTGCCAGTTTCG-3', HER4 reverse: 5'-GGGAGGCCAGCATCGTGTA-3'; GAPDH forward: 5'-TGCCCAGAA CATCAT CCCT-3', GAPDH reverse: 5'-GTCCTCAGTGL AGCCCAAG-3'.

### Tumor xenografts

Twenty female BALB/c mice, ageing 4-6 weeks, were purchased from the Shanghai Laboratory Animal Center (Shanghai, China). The animals were randomly divided into two groups. Mice were seeded in a pathogen-free environment, kept under a 12 h-light/dark cycle and with free access to water and food. The body weight of each mouse and the dimensions (length and width) of tumors were monitored every 3 days. Animal care protocols and experiments were approved by the animal ethics committee of Luoyang Orthopaedic Hospital of Henan Province and Orthopaedic Hospital of Henan Province.

### Immunohistochemistry

The tumor slices were heated overnight at 60°C and then incubated with the indicated antibodies at 4°C overnight and the appropriate secondary antibodies for 30 min at room temperature. The images were observed using an Olympus light microscope.

### Statistical analysis

All data are presented as the mean±standard deviation. Student's t-tests were used to assess the differences between groups. Statistical analyses were performed using the SPSS version 16.0 software (SPSS Inc., Chicago, IL, USA). P-values <0.05 denoted statistically significant differences.

## Results

### 1. HER4 was upregulated in osteosarcoma tissues and positively correlated with poor survival

Immunohistochemistry (IHC) analysis was used to determine the localization and expression of HER4 in 75 osteosarcoma samples and normal adjacent bone tissues. As shown in Fig. 1A, HER4 was positively expressed in the cytoplasm of osteosarcoma specimens. The positive expression rate of HER4 in osteosarcoma samples was significantly higher than that recorded in adjacent tissue samples. The Kaplan-Meier plotter was used to detect the prognostic value of HER4 expression in patients with osteosarcoma. The data showed that patients with higher HER4 expression had significantly shorter OS than others (P<0.05) (Fig. 1B). This finding is consistent with the disease-free survival results, indicating that HER4 expression may have prognostic significance in osteosarcoma.

Subsequently, the correlation between HER4 expression and different clinicopathological factors in osteosarcoma was analyzed. As shown in Table 1, there was no significant association noted between HER4 and sex, age, tumor size, or histological grade (all P>0.05). However, the levels of HER4 were positively correlated with high Enneking stage, lung metastasis, and recurrence (all P<0.05).

qRT-PCR and western blotting were used to measure the mRNA and protein levels of HER4, respectively, in osteosarcoma cell lines. As shown in Fig. 1C, the protein levels of HER4 were elevated in U2OS, MG-63, Saos2, and HOS cells compared with those detected in human hFOB1.19 cells (P<0.05) (Fig. 1C). However, the mRNA levels of HER4 in U2OS and MG-63 cells were significantly higher than those measured in SaoS2 and HOS cells (P<0.05) (Fig. 1D).

Therefore, U2OS and MG-63 cells were selected for subsequent experiments.

Moreover, Univariate Cox regression and multivariate Cox regression analyses showed that recurrence, lung metastasis, and high HER-4 expression were independent predictors of poor OS (Table 2).

### 2. HER4 knockdown inhibited cell proliferation and facilitated osteosarcoma invasion/migration and EMT

To clarify the role of HER4 in the development of osteosarcoma,three shRNA sequences were designed and used to downregulate the levels of HER4. Sh-HER4#1, sh-HER4#2, sh-HER4#3, or the sh-control was transfected into U2OS and MG-63 cells. The results suggested that the mRNA and protein expression of HER4 was obviously downregulated by sh-HER4-1#, sh-HER4-2#, and sh-HER4#3 after 48 h (Figs. 2A, 2B). Moreover, the inhibitory effect of sh-HER4#1 was higher than that of the others (P<0.05). Therefore, sh-HER4#1 was selected for subsequent experiments.

As shown in Fig. 2C, MTT assay was used to observe the effect of HER-4 on osteosarcoma cells proliferation.Compared with sh-con groups, sh-HER4 markedly decreased U2OS and MG-63 cell viability (P<0.05). A colony formation assay was also carried out to assess the cell proliferation (Figs. 2D, 2E). HER4 knockdown suppressed colony formation (P<0.05), indicating that HER4 expression promotes the viability of MG-63 and U2OS cells.

Invasion and migration play key roles in cancer progression. To determine whether HER-4 was related to the migration/invasion of osteosarcoma cells, Transwell assays and wound closure analysis were used respectively. As shown in Fig. 2F-2G, sh-HER4 significantly suppressed the invasive ability of U2OS and MG-63 cells (P<0.05). Similarly, HER-4 knockdown significantly inhibited cell migration compared to controls (Fig. 2H, 2I).

EMT is a dynamic biological process that ultimately leads to metastasis and stemness maintenance 22. Consistent with the results of the invasion/migration experiments, HER4 knockdown reduced the levels of matrix metalloproteinase 2 (MMP2), α-SMA, and vimentin, whereas it increased those of E-cadherin in U2OS and MG-63 cells (Figs. 2J, 2K).

### 3. HER4 increased stemness properties and CD133+ subpopulations in osteosarcoma cells

Spheroid formation assays were performed to evaluate the effects of HER4 on the self-renewal ability of cells. HER4 knockdown reduced the number and volume of spheroids on ultra-low-attachment plates (Figs. 3A, 3B). Notably, HER4 knockdown also decreased the CD133+ subpopulation of cells (Figs. 3C, 3D), and reduced the expression of stemness markers SOX2, NANOG, and Oct4 (Figs. 3E, 3F).

### 4. The PI3K/AKT pathway facilitated the HER4-mediated regulation of U2OS and MG-63 cell invasion/migration

As shown in Figs. 4A and 4B, HER4 knockdown markedly attenuated p-PI3K and p-AKT S473 expression. This finding indicated that the PI3K/mTOR signaling pathway may participate in the HER4-mediated modulation of osteosarcoma progression. The specific inhibitor LY294002, which also effectively inhibits AKT S473 phosphorylation, was added to further investigate the role of the PI3K/mTOR signaling pathway. As shown in Fig. 4C, sh-HER4 markedly reduced cell proliferation compared with the sh-control group. Notably, pretreatment with LY294002 further decreased proliferation (P<0.05) in the LY294002+sh-HER4 group. Similarly, LY294002 significantly aggravated the sh-HER4-inhibited invasion/migration of U2OS and MG-63 cells (Figs. 4D-4G). Smaller spheroid volumes and fewer CD133-positive cells were detected in the LY294002+sh-HER4 group (Figs. 4H-4K). Taken together, these findings indicate that HER4 regulates the development and stemness traits of osteosarcoma via the PI3K/mTOR pathway.

### 5. HER4 regulates the PTEN-dependent progression of osteosarcoma through the PI3K/AKT pathway

The PTEN-PI3K/AKT axis negatively regulates the progression of hepatocellular carcinoma, breast cancer, and pancreatic cancer. As shown in Fig. 5A, we found that sh-HER4 markedly increased the levels of p-PTEN. Moreover, sh-PTEN significantly increased the protein levels of p-PI3K and p-AKT, and reversed the sh-HER4-mediated downregulation of p-PI3K and p-AKT expression (Fig. 5B). These results indicated that PTEN plays a pivotal role in the HER4-mediated progression of osteosarcoma via the PI3K/AKT pathway.

As shown in Fig. 5C, compared with control group, cell viability of sh-PTEN group was sightly upregulated; and sh-PTEN partly offseted the inhibitory effect of sh-HER-4 on cell proliferation (P<0.05). sh-PTEN further rescued the sh-HER4-mediated reduction in cell invasion and wound closure (Figs. 5D-5G). In addition, smaller spheroid volumes and fewer CD133-positive cells were detected in the sh-PTEN+sh-HER4 group (Figs. 5H-K). Collectively, these findings indicate that HER4 regulates the progression and stemness traits of osteosarcoma via the PTEN/PI3K/mTOR pathway.

### 6. Knockdown of HER4 inhibits tumorigenicity *in vivo*

As shown in Fig. 6A and 6B, the tumors derived from the HER-4 shRNA group were significantly smaller in size and much lighter in weight compared withsh-control group. IHC staining was used to examine the expression of p-PI3K and p-AKT in xenograft tumors. As shown in Fig. 6C, HER-4 shRNA group exhibited significantly faded p-PI3K and p-AKT levels, as well as increased p-PTEN expression.

As we have confirmed that HER-4 played the positive role in cell invasion/migration *in vitro* experiments. To substantiate these observations *in vivo* experiments, lung tissues were taken from the sacrificed mice, then H&E staining was used. As shown in Fig. 6D, sh-HER-4 treatment resulted in less lung metastatic lesions than those observed in the control group. All the above data indicated that HER-4 promoted tumorigenesis in osteosarcoma cells through PTEN/PI3K pathway.

## Discussion

Hyperactivation of ErbB family members, including HER4, promotes the development and progression of osteosarcoma, and is linked to poor prognosis 23. However, few studies have investigated the effects of HER4 on the progression of osteosarcoma. Wang *et al* reported constitutive HER4 phosphorylation in early-passage osteosarcoma cells 13; however, this was only associated with distant metastasis (P<0.05) and not related to sex, age, tumor location, histological subtype, or surgical stage. Another study found that HER4 was not positively correlated with clinicopathological features of patients with osteosarcoma (P>0.05). Thus, the results of these previous studies are unilateral and fragmentary.

IHC staining results and statistical analysis indicated that HER4 expression was not associated with sex, age, tumor size, tumor location, or histological grade (P>0.05); however, it was strongly positively correlated with high Enneking stage, lung metastasis, and recurrence, in contrast to the findings reported by Wang *et al* 13. In addition, both overall survival and progression-free survival were shorter in osteosarcoma patients with higher expression of HER4. Moreover, the levels of HER4 in U2OS, MG-63, and HOS cells were variously elevated compared with those measured in hFOB1.19 cells (P<0.05). All the above results support previous suggestions that HER4 represents a prognostic factor for osteosarcoma.

Although several studies have shown that knockdown of HER4 suppresses the proliferation and anchorage-independent growth of osteosarcoma cells, it was unclear whether HER4 modulates the invasion/migration of these cells. As shown in Figs. 2A-C, sh-HER4 markedly attenuated the proliferation of U2OS and MG-63 cells and colony formation. Shi *et al* showed that ETS homologous factor promoted invasion/migration by modulating HER2-4 24. In the present study, sh-HER4 reduced the number of invasive cells (Figs. 2F, 2G) and delayed wound closure (Figs. 2H, 2I), in addition to attenuating the EMT phenotype (Figs. 2J, 2K). This is the first evidence to demonstrate that HER4 promotes cell invasion/migration and EMT in osteosarcoma. Also, EMT has been linked to the acquisition of stem cell-like properties by cancerous cells 25. Wang *et al* reported that ErbB signaling promoted EMT and cancer stem cell-like traits in prostate cancer cells 26. Parris *et al* found that overexpression of erbB-2 facilitated the stemness of breast cancer cells 27. Consistent with the above findings, we observed that knockdown of HER4 led to a smaller spheroid size, decreased CD133+ ratio, and reduced expression of stemness markers (Fig. 3).

In addition, PTEN may negatively regulate the PI3K/AKT pathway to modulate cell proliferation, invasion/migration, and tumorigenesis in osteosarcoma 28-29. Furthermore, the PTEN/PI3K/AKT pathway promotes maintenance of stemness in liver, lung, and breast cancers, as well as in chronic myeloid leukemia 30-33. In the present study, HER4 knockdown elevated the levels of PTEN and downregulated the expression of p-PI3K and p-AKT.

These findings indicated that HER4 regulated the progression of osteosarcoma via the PTEN/PI3K/AKT pathway. Pretreatment with the specific PI3K inhibitor LY294002 enhanced the sh-HER4-induced inactivation of the PI3K/AKT pathway, suppression of proliferation, invasion, and wound closure, and reduction in spheroid size and number of CD133-positive cells. In contrast, sh-PTEN reversed the sh-HER4-mediated downregulation of p-PI3K and p-AKT stemness-related markers, expression of EMT-related markers, proliferation, invasion, wound closure, spheroid size, and number of CD133-positive cells. Sh-HER4 also reduced the tumor size and decreased the expression of p-PI3K, p-AKT, p-PTEN, and MMP2 in mouse tissue (Fig. 6). The results demonstrate that HER4 mediates the PTEN-dependent proliferation, invasion/migration, and stemness maintenance of osteosarcoma cells via the PI3K/AKT pathway.

In conclusion, our research provide strong evidence for the first time that HER4 promotes tumorigenesis and the development of osteosarcoma by enhancing the invasion/migration and stemness features through the PTEN/PI3K-AKt signaling. However, based on the finding of this study, HER4 is a potential biomarker and therapeutic target for osteosarcoma.

## Figures and Tables

**Figure 1:** HER4 expression in both osteosarcoma specimens and cell lines. (A) HER4 expression in osteosarcoma specimens and normal adjacent tissues, detected by immunohistochemical analysis. (B) Kaplan-Meier curves for the assessment of survival. The relationship between the survival rate of patients with osteosarcoma and the expression of HER4 was analyzed. (C) Protein levels of HER4 in osteosarcoma cell lines. (D) The mRNA expression of HER4 in osteosarcoma cell lines. *P<0.05

**Figure 2:** sh-HER4 suppressed cell proliferation and invasion/migration. (A) qRT-PCR was used to detect the knockout efficiency of HER4. (B) Western blotting was performed to investigate the knockout efficiency of HER4. (C) MTT cell viability assay. (D, E) Colony formation assay for U2OS and MG-63 cells. (F, G) HER4 knockdown reduced the invasive ability of U2OS and MG-63 cells (magnification: 200×). (H, I) sh-HER4 delayed wound closure of U2OS and MG-63 cells. Right panels, quantitative data. (J, K) Protein expression of E-cadherin, vimentin, α-SMA, and MMP2 in MG-63 and U2OS cells treated with or without sh-HER4. GAPDH was used as a loading control. Data are expressed as the mean±SD of three independent experiments. *P<0.05 vs. sh-control group.

**Figure 3:** sh-HER4 blocked the stemness and enriched the CD133+ subpopulations of osteosarcoma cells. (A, B) Transfected with sh-HER4 shrinked the scale of spheroids of of U2OS and MG-63 cells. Representative images (left panel) and statistical measurements (right panel). Representative micrographs of spheres formed in cells. Scale bar: 100 μm. (C, D) Percentage of CD133+ cells in U2OS- and MG-63-derived spheroids as analysised by flow cytometry. (E, F) Western blotting was performed to measure the protein expression of stem cell-associated genes. *P<0.05 vs. sh-control group.

**Figure 4:** The role of HER4 in the PI3K/mTOR signaling pathway. (A, B) The western blotting was used to measure the protein expression of phophorylated PI3K (p-PI3K), p-AKT, and p-PTEN. (C) The cell viability was assessed by MTT assay.(D, E) Transwell assay was carried out to determine the invasive ability of cells. (F, G) Wound healing assay was performed to measure the migration ability of cells. (H,I)Spheroid formation assay for U2OS and MG-63 cells transfected with sh-HER4 with or without LY294002 pretreatment. Representative images (left panel) and statistical measurements (right panel). (J, K) The flow cytometry was used to determine percentage of CD133+ cells in U2OS- and MG-63-derived spheroids.*P<0.05 vs. sh-control group; ^&^P<0.05 vs. LY294002 group.

**Figure 5:** PTEN facilitated the HER4-mediated regulation of osteosarcoma progression. (A) Phosphorylated-PI3K (p-PI3K), p-AKT, and p-PTEN expression as measured by western blotting analysis. (B) Western blotting analysis of p-PI3K, p-AKT, and p-PTEN. (C) MTT assay for the analysis of cell viability after transfection with sh-HER4 with or without sh-PTEN pretreatment. (D, E) Transwell assay to determine the invasive ability of cells. (F, G) Wound healing assay to record the migratory ability of cells. (H, I) Spheroid formation assay for U2OS and MG-63 cells transfected with sh-HER4 with or without sh-PTEN pretreatment. Representative images (left panel) and statistical measurement (right panel). (J, K) Percentage of CD133+ cells in U2OS- and MG-63-derived spheroids, as determined by flow cytometry. *P<0.05 vs. si-control group; ^&^P<0.05 vs. si-PDK1 group.

**Figure 6:** HER4 contributed to tumorigenicity *in vivo*. (A and B) Images of xenograft tumors formed in nude mice with shRNA silencing of HER4 and sh-control cells (negative control). The volume and weight of xenograft tumors are summarized. (C) Representative images of IHC expression of phosphorylated-PTEN (p-PTEN), p-PI3K, and p-AKT in tumor nodules. *P<0.05 vs. sh-control group. (D) Histological figures of pulmonary metastases in nude mice. HER4, human epidermal growth factor receptor 4; IHC, immunohistochemistry; PTEN, phosphatase and tensin homolog; shRNA, short hairpin RNA.

**Table 1:** The relationship between HER-4 expression and pathological characteristics.

Characteristics	HER-4						
	+		-		X2	P	
Gender				3.406			0.065
Male	23	18					
Female	26	8					
Age(year)				1.422			0.2333
>18	25	15					
<18	24	11					
Lung metastasis				6.039			0.014*
yes	6	12					
NO	43	14					
Tumor size(d/cm)				0.126			0.723
>5	30	17					
<5	19	9					
Ennecking stage				9.228			0.002*
IIA	19	20					
IIB	21	5					
III	9	1					
Histological type				4.22			0.057
Osteoblastic	8	12					
Chondroblastic	18	8					
Fibroblastic	23	6					
Recurrence				5.802			0.016*
Yes	33	24					
No	16	2					
							

**Table 2:** Cox regression analysis for overall survival.

Characteristics	Univariate analysis			Multivariate analysis		
	HR	95% CI	P-value	HR	95% CI	P-value
Gender						
Female vs male	1.124	(0.912-1.547)	0.142			
Years						
>18 vs <18	0.974	(0.748-1.254)	0.368			
Ennecking stage						
II vs I	3.521	(1.406-8.818)	0.000*	3.005	(1.327-6.805)	0.000*
III vs II	3.796	(2.613-5.515)	0.000*	2.504	(1.425-4.400)	0.003*
Tumor size						
>5 vs <5	1.399	(0.951-2.058)	0.323			
Recurrence						
Yes vs No	2.102	(1.574-3.847)	0.004*	1.547	(1.327-3.874)	0.028*
Lung metastasis						
Yes vs No	1.748	(1.254-4.4012)	0.013*	1.857	(1.104-4.12)	0.007*
